RETRACTED

# Computational Prediction of Intrinsically Disordered Proteins Based on Protein Sequences and Convolutional Neural Networks

**DOI:** 10.1155/2021/4455604

**Published:** 2021-12-28

**Authors:** Hao He, Yong Yang

**Affiliations:** ^1^School of Electronic and Information Engineering, Hebei University of Technology, Tianjin 300401, China; ^2^School of Computer Science and Technology, Tiangong University, Tianjin 300387, China

## Abstract

Intrinsically disordered proteins (IDPs) possess at least one region that lacks a single stable structure in vivo, which makes them play an important role in a variety of biological functions. We propose a prediction method for IDPs based on convolutional neural networks (CNNs) and feature selection. The combination of sequence and evolutionary properties is used to describe the differences between disordered and ordered regions. Especially, to highlight the correlation between the target residue and adjacent residues, multiple windows are selected to preprocess the protein sequence through the selected properties. The shorter windows reflect the characteristics of the central residue, and the longer windows reflect the characteristics of the surroundings around the central residue. Moreover, to highlight the specificity of sequence and evolutionary properties, they are preprocessed, respectively. After that, the preprocessed properties are combined into feature matrices as the input of the constructed CNN. Our method is training as well as testing based on the DisProt database. The simulation results show that the proposed method can predict IDPs effectively, and the performance is competitive in comparison with IsUnstruct and ESpritz.

## 1. Introduction

Intrinsically disordered regions (IDRs) of proteins often play an important role in many biological functions while lacking a single stable structure in vivo [1]. Intrinsically disordered proteins (IDPs) can be fully or partially unstructured and generally include one or more IDRs [2]. IDPs are very common in eukaryotes. They carry out many important functions such as cell signaling and translation and can promote molecular recognition as well as protein-protein interactions [3]. Many functions of IDPs are directly associated with their structural attributes [4]. Moreover, previous studies have shown that IDPs are key players in human disease [5]. For example, 79% of cancer-related proteins are IDPs and 57% of cardiovascular disease-related proteins are IDPs [6, 7]. Besides, IDPs are also correlated with genetic diseases, neurodegenerative diseases, and Alzheimer's disease [8, 9]. Therefore, accurate prediction of IDPs is not only important for protein description and functional annotations but also contributing to the drug design.

RETRACTED

There are a lot of experimental techniques for identifying IDPs, such as X-ray crystallography, nuclear magnetic resonance (NMR), and circular dichroism (CD) spectroscopy. However, the experimental methods are expensive and time-consuming due to the difficulty of purification and crystallization [10]. Therefore, it is necessary to predict IDPs based on computational methods.

During the past decade, many computational methods are proposed for the prediction of IDPs. These methods can be roughly divided into three categories [11]. (1) Physicochemical-based methods: these methods are based on physicochemical properties and propensity scales of amino acids, such as FoldIndex [12], GlobPlot [13], and IsUnstruct [14]. FoldIndex predicts IDPs by calculating the ratio of average hydrophobicity to average net charge of protein sequences. GlobPlot establishes a mapping scale to reflect the relative tendency of each amino acid residue in the ordered or disordered state based on the probability of each amino acid being in a regular secondary structure or random curl and predicts IDPs through a kernel function and filter. IsUnstruct uses the Ising model to describe the interaction between ordered and disordered states and achieves good performance. Thus, we select it as one of comparison methods. (2) Machine learning-based methods: these methods treat IDPs prediction as a binary classification problem that use positive and negative samples to distinguish ordered and disordered residues. Commonly used classification algorithms include neural network (NN), radial basis function network (RBFN), support vector machine (SVM), random forest, and so on. The representative methods in this category contain DisPSSMP [15], Dispredict [16], SPINE-D [17], ESpritz [18], RFPR-IDP [19], and so on. DisPSSMP combines RBFN and a matrix PSSMP to predict IDPs. The matrix PSSMP is a condensed position-specific scoring matrix (PSSM) according to different physicochemical properties. Dispredict uses three kinds of features which include sequence information, evolutionary information, and structural information and predicts IDPs based on SVMs with Radial Basis Function kernel. SPINE-D is based on NN with two-hidden-layer neural network and an additional one-layer filter for smoothing prediction results. ESpritz is an ensemble of three NNs for predicting the N-terminal, internal, and C-terminal of proteins, respectively. Based on bidirectional recursive neural network, it achieves good prediction performance. Thus, it is also selected as a comparison method. (3) Meta methods: these methods combine various prediction methods into one model to further improve the prediction performance, such as MetaDisorder [20], DisCop [21], and MobiDB-lite [22]. MetaDisorder has 13 independent predictors. The final prediction result of MetaDisorder is obtained by the weighted value of the results of these 13 predictors. It possesses high prediction accuracy, but the operation is slow because it contains so many independent predictors. DisCop uses a rational design to construct a metapredictor, which selects the best performance set of 6 predictors from 20 basic predictors. The prediction results of these methods are then combined by using a regression model. MobiDB-lite is constructed based on 8 predictors, whose final consensus prediction is determined by voting.

RETRACTED

In this paper, we propose a method to predict IDPs based on CNN and feature selection. Considering that CNN has achieved very good results in computer vision, natural language processing, and other fields, we expect to extract more hidden features by using CNN. Our previous work [23] confirms this expectation. In this paper, we improve the preprocessing process and reconstruct and train the CNN and further improve the prediction performance. The input features include sequence properties and evolutionary properties. Moreover, to highlight their specificity, sequence and evolutionary properties are preprocessed by multiple windows, respectively. Then, the preprocessed features are combined into a feature matrix as the input of the prediction model. Through preprocessing, the input information can reflect the relationships between each feature and its neighboring features in the feature matrix and enrich the feature information extracted from protein sequences. Our prediction model contains two convolutional layers and one fully connection layer and is trained and tested on the DisProt database [24]. Finally, the proposed method is compared with two competitive prediction methods IsUnstruct and ESpritz based on the same test set.

## 2. Materials and Methods

We select 12 sequence properties and 20 pieces of evolutionary properties. The two kinds of properties are preprocessed, respectively, to highlight their specificity. Then, we train a CNN model which includes two convolutional layers and one fully connected layer to predict IDPs.

### 2.1. Dataset

The DisProt database is used to train and test the proposed methods. There are 803 protein sequences, which contain 1,254 disordered regions and 1,343 ordered regions, corresponding to 92,418 disordered residues and 315,856 ordered residues, respectively. The 803 protein sequences are randomly divided into two subsets according to the ratio of 9 : 1. The large dataset is the training set, containing 721 sequences with 85,184 disordered residues and 289,983 ordered residues. The small dataset is the test set, containing 82 sequences with 7,234 disordered residues and 25,873 ordered residues.  Table 1 lists the specific information.

RETRACTED

### 2.2. Selected Properties

Since the complexity of the protein sequence denotes how it can be rearranged in different ways, the low complexity regions are more likely to be disordered than ordered. We select five complexity features discussed in our previous work [25], which include topological entropy, Shannon entropy, and three amino acid propensities. Among these features, topological entropy may not be calculated directly from the protein sequence because the sequence contains 20 amino acids elements and the length of sequence does not satisfy the conditions for calculating topological entropy. Thus, before calculating the topological entropy, we map the protein sequence to 0-1 sequence. Considering the characteristics of disordered residues, large hydrophobic amino acid residues (I, *L*, and V) and aromatic amino acid residues (F, W, and Y) are mapped to 1, and other residues are mapped to 0. Given a protein region {*w*(*j*), 1 ≤ *j* ≤ *N*} of length *N*, its topological entropy *H*_*T*_(*w*) can be calculated as follows:

(1) $$\begin{array}{c} H_{T}\left(w\right)=\;\frac{1}{N-\left(2^{n}+n-1\right)+1}\overset{N-\left(2^{n}+n-1\right)+1}{\underset{l=1}{\sum }}\frac{\log_{2}p_{w_{l}^{2^{n}+n-1+l-1}}\left(n\right)}{n}, \end{array}$$

where *p*_*w*_*l*_^2^*n*^+*n*−1+*l*−1^_(*n*) denotes the number of different subsequences with length of *n* in the region *w*(*l*) ⋯ *w*(2^*n*^+*n* − 1). The length of subsequences *n* satisfies the following:

(2) $$\begin{array}{c} 2^{n}+n-1\leq \left|w\right|<2^{n+1}+\left(n+1\right)-1. \end{array}$$

For the same protein region *w*, the Shannon entropy *H*_*S*_(*w*) can be described as follows:

(3) $$\begin{array}{c} H_{S}\left(w\right)=-\sum_{k=1}^{20}f_{k}\log_{2}f_{k}, \end{array}$$

where *f*_*k* _(1 ≤ *k* ≤ 20) is the probability of 20 amino acids appearing in the region *w*.

Three amino acid propensities are selected from GlobPlot [13], which contain Remark 465, Deleage/Roux, and Bfactor (2STD). For these three propensities, the protein region *w* is mapped to them, and then the average values of the mapped regions are calculated as follows:

(4) $$\begin{array}{c} m_{p}\left(w\right)=\left[m_{p1}\left(w\right),m_{p2}\left(w\right),m_{p3}\left(w\right)\right]=\frac{1}{N}\sum_{l=1}^{N}w^{pi}\left(l\right),\;\;i=1,2,3. \end{array}$$

In (4), the parameter *w*^*pi*^ represents the mapped region of *w* with the *i*-th propensity, where *i*=1,2,3 correspond to Remark 465, Deleage/Roux, and Bfactor, respectively.

RETRACTED

In addition, it has been demonstrated that disordered regions and ordered regions usually show different physicochemical properties, and thus physicochemical properties are very useful in IDPs prediction. We select seven commonly used physicochemical properties, which is collected by Jens et al [26]. They are steric parameter, polarizability, volume, hydrophobicity, isoelectric point, helix probability, and sheet probability. Following that, the average value of the mapped target region is calculated:

(5) $$\begin{array}{c} m_{a}\left(w\right)=\left[m_{a1}\left(w\right),\cdots ,m_{ai}\left(w\right),\cdots m_{a7}\left(w\right)\right]=\frac{1}{N}\sum_{l=1}^{N}w^{ai}\left(l\right). \end{array}$$

Similar to (4), the parameter *w*^*ai*^ in (5) represents the mapped region of *w* with the *i*-th physicochemical properties and *i*=1,2, ⋯, 7.

Finally, the PSSM is used to describe the evolutionary of each protein sequence as the evolutionary properties to enrich the information of protein sequences. They are obtained by performing three iterations of PSI-BLAST (Position-Specific Iterative Basic Local Alignment Search Tool) on NCBI (National Center for Biotechnology Information) nonredundant database with default parameters. For a protein sequence with length *L*, a *L* × 20 matrix *M*_*pssm*_*L*_ can be obtained. Then, the evolutionary properties of the region intercepted by the window of length *N* can be expressed by a *N* × 20 matrix *M*_*pssm*_*w*_.

### 2.3. Preprocessing

In order to highlight their specificity, sequence and evolutionary properties are preprocessed, respectively. Given a protein sequence of length *L*, we select a window of length *N* and append N/2 zeros to both ends of the protein sequence. For sequence properties, each region is intercepted by the window, and a 12 dimensional vector *v*_*i*_(1 ≤ *i* ≤ *L*) can be calculated by the following:

(6) $$\begin{array}{c} v_{i}={\left[H_{T}\left(w\right),\;H_{S}\left(w\right),\;m_{p}\left(w\right),\;m_{a}\left(w\right)\right]}^{T}. \end{array}$$

Assign *v*_*i*_ to each residue in the *i*-th window. Sliding the window, each residue is associated with multiple *v*_*i*_. For each residue, the sequence feature vector *x*_*j*_^*seq*^(1 ≤ *j* ≤ *L*) is the average of all *v*_*i*_ about it, which can be described as follows:

(7) $$\begin{array}{c} x_{j}^{seq}=\left\{\begin{array}{cc} \frac{1}{j+N_{0}}\sum_{i=1}^{j+N_{0}}v_{i}, & 1\leq j\leq N_{0},\\ \frac{1}{N}\sum_{i=j+N_{0}-N+1}^{j+N_{0}}v_{i}, & N_{0}<j\leq L-N_{0},\\ \frac{1}{L_{0}-j-N_{0}+1}\sum_{i=j+N_{0}-N+1}^{L_{0}-N+1}v_{i}, & L-N_{0}<j\leq L. \end{array}\right. \end{array}$$

In (7), *X*_*j*_=[*x*_*j*_^1^ *x*_*j*_^2^ ⋯ *x*_*j*_^*n*_*win*_^ ⋯ *x*_*j*_^*N*_*win*_^], and *X*_*j*_=[*x*_*j*_^1^ *x*_*j*_^2^ ⋯ *x*_*j*_^*n*_*win*_^ ⋯ *x*_*j*_^*N*_*win*_^] denotes the sequence length after appending zeros.

RETRACTED

For evolutionary properties, each region is intercepted by the window gets a *N* × 20 matrix *M*_*pssm*_*w*_. We calculate the average value of the matrix of the intercepted region and obtain a 20 dimensional vector which is served as the evolutionary feature vector *x*_*j*_^*evo*^(1 ≤ *j* ≤ *L*) for the central residue in the region:

(8) $$\begin{array}{c} x_{j}^{evo}={\left(\frac{1}{N}\sum_{l=1}^{N}M_{pssm\_w}\left(l,1:20\right)\right)}^{T}. \end{array}$$

Then, for each residue, a 32-dimensional feature vector *x*_*j*_=[*x*_*j*_^*seq*^; *x*_*j*_^*evo*^] can be obtained.

In this paper, we select multiple windows to perform the preprocessing. According to the preprocessing, each residue can get a 32-dimensional feature vector *X*_*j*_=[*x*_*j*_^1^ *x*_*j*_^2^ ⋯ *x*_*j*_^*n*_win_^ ⋯ *x*_*j*_^*N*_win_^] for each window, where *X*_*j*_=[*x*_*j*_^1^ *x*_*j*_^2^ ⋯ *x*_*j*_^*n*_win_^ ⋯ *x*_*j*_^*N*_win_^] denotes the label of the window. Then, the feature vectors calculated by different windows are combined into a feature matrix. Assuming that the number of selected windows is *X*_*j*_=[*x*_*j*_^1^ *x*_*j*_^2^ ⋯ *x*_*j*_^*n*_win_^ ⋯ *x*_*j*_^*N*_win_^], the feature matrix of each residue *X*_*j*_=[*x*_*j*_^1^ *x*_*j*_^2^ ⋯ *x*_*j*_^*n*_win_^ ⋯ *x*_*j*_^*N*_win_^] can be expressed as follows:

(9) $$\begin{array}{c} X_{j}=\left[x_{j}^{1}\;x_{j}^{2}\cdots x_{j}^{n_{\text{win}}}\cdots x_{j}^{N_{\text{win}}}\right]. \end{array}$$

So, each residue can obtain a feature matrix of 32 × *N*_win_, where each row represents the preprocessing results of a certain feature at different windows and each column represents the preprocessing results of 32 features at a certain window. Thus, there are some correlations between the rows and columns of the feature matrix.

### 2.4. Designing and Training the CNN

We design a convolutional neural network (CNN) with two convolutional layers as well as one fully connected layer, and each convolutional layer is followed by a pooling layer, as shown in Figure 1. Since the scale of the feature matrix calculated is small, the convolution kernels are set to small scales when the CNN is designed. At the same time, because of the large number of learning samples, fewer convolution kernels and convolutional layers are selected to simplify the operation.

In the network, the activation functions of the convolutional layers are ReLu functions and the activation functions of the output layer are softmax functions. The parameters of the first convolutional layer (conv1) are set to 3 × 3 × 1 × 8 preliminarily, where 3 × 3 is the size of the convolution kernel, and 1 denotes the number of channels and 8 denotes the number of convolution kernels. Similarly, the parameter of the second convolutional layer (conv2) is 2 × 2 × 8 × 8. In each convolutional layer, the convolution step is 1 and performs same padding with zero. The two pooling layers use max pooling with 2 × 2 filters.

RETRACTED

In the designed CNN, the gradient descent algorithm is replaced by the Adam algorithm in the backward propagation to update parameters. In order to improve the operation speed, minibatch is used to update parameters. That is, the sample set is divided into multiple subsets of equal scale for each iteration, and each subset is used to calculate the gradient and update the parameters one by one. Finally, combined with the feature selection and extraction, Figure 2 shows the prediction procedure of the proposed method.

## 3. Results and Discussion

### 3.1. Performance Evaluation

Four metrics are used to evaluate the proposed method, which include sensitivity (Sens), specificity (Spec), weighted score (Sw), and Matthews correlation coefficient (MCC). The Sw and MCC can be computed as follows:

(10) $$\begin{array}{c} \text{Sw}=\text{Sens}+\text{ Spec,}\\ \text{MCC}=\frac{\left(\text{TP}\times \text{TN}\right)-\left(\text{FP}\times \text{FN}\right)}{\sqrt{\left(\text{TP}+\text{FP}\right)\left(\text{TP}+\text{FN}\right)\left(\text{TN}+\text{FP}\right)\left(\text{TN}+\text{FN}\right)}}. \end{array}$$

where Sens=TP/(TP+FN), Spec=TN/(TN+FP), and TP, TN, and FN as well as FP are corresponding to the number of true positives, true negatives, false negatives, and false positives.

### 3.2. Impacts of Different Number of Windows

The lengths of windows are selected in the interval of [7, 55] firstly. The odd numbers in the interval are selected as the window lengths, which is [7, 9,…, 55]. Then, starting from the length of 7, we increase the step length from 1 to 4 to select windows, and thus the numbers of selected windows are 25, 13, 9, and 7, respectively. At this point, the parameters of conv1 and conv2 are set to 3 × 3 × 1 × 8 and 2 × 2 × 8 × 8, respectively. The 2 × 2 filters are used in the pooling layers to perform max pooling. The learning rate is 0.005.  Table 1 and Figure 3 show the prediction results of 10-fold cross validation on the training set with different number of windows.

From Table 2, with the decrease in the number of windows, the value of Sens fluctuates and the value of Spec has an upward trend. And at the same time, the values of Sw and MCC increase with the decrease in the number of windows, as shown in Figure 3. Since the number of windows is inversely proportional to the distance between windows, when the window distance is small, that is, the number of windows is large, the redundancy of the calculated feature matrix is relatively high, and the prediction performance is damaged.

RETRACTED

Considering that the prediction result of *N*_*win*_=7 is similar to *N*_*win*_=9, we add some longer windows to them and make the length of the longest window around 90. In the case of *N*_*win*_=7, the set of window is [7, 15,…, 55]. We increase the number of windows by the distance between them which is equal to 8. Then, the window data set becomes [7, 15,…, 87] and *N*_*win*_=11. Similarly, in the case of *N*_*win*_=9, the set of window [7, 13,…, 55] is increased to [7,13,…, 91], and the number of windows in the new set is *N*_*win*_=15. The prediction results of them are shown in Table 3.

From Table 3, adding some longer windows can improve the value of Sw. And the Sw of *N*_win_=11 and *N*_win_=15 is similar. However, the MCC of *N*_*win*_=11 is much larger than that of *N*_win_=15, so we choose the windows in *N*_win_=11, that is, [7, 15,…, 87].

### 3.3. Impacts of Different Number of Convolutional Layers

Our CNN model is designed by several submodules which contain a convolutional layer and a pooling layer. Thus, when we add a convolutional layer, it is followed by a pooling layer. In this section, we add convolutional layers on the basis of the network structure in Figure 2, which includes 2 convolutional layers. For all the additional convolutional layers, the parameter is set to 2 × 2 × 8 × 8.  Table 4 shows the prediction results of 10-fold cross validation on the training set with different convolutional layers.

In Table 4, with the increase in the number of layers, although the values of Spec fluctuated, the values of Sens show downward trend and the values of Sw and MCC also show downward trend. Therefore, we still use two convolutional layers in the prediction model.

### 3.4. Impacts of Different Scales of Convolution Kernels

We change the scale of convolution kernels to analyze the influence on the prediction performance. Firstly, the number of convolution kernel in conv1 is set to 8, and the parameter of the second convolution layer conv2 is 2 × 2 × 8 × 8. At the same time, the scale of the convolution kernel in conv1 is changed as shown in Table 5. Since the scale of feature matrix is only 32 × 11, the scale of convolution kernel should not be too large. We select four scales for comparison. Table 5 shows the prediction results of 10-fold cross validation on the training set with different convolution kernels in conv1. Although kernel of 2 × 2 gets the highest Sens and kernel of 4 × 4 gets the highest Spec, these four scales of convolution kernel obtain similar Sw and MCC. Considering that the Sw of kernel of 2 × 2 is slightly higher than others, we finally set the convolution kernel of conv1 to 2 × 2.

RETRACTED

After determining the scale of convolution kernel in conv1, we change the scale of convolution kernel in conv2. In this case, the parameter of conv1 is 2 × 2 × 8 × 8. Similar to the selection of conv1, we also compare the same four scales for conv2. The predicted results are shown in Table 6.

The convolution kernels of 5 × 5 and 3 × 3 obtain the highest Sens and Spec, respectively. However, the kernel of 2 × 2 possesses much better Sw. Therefore, the scale of convolution kernel in conv2 is set to 2 × 2.

### 3.5. Impacts of Different Number of Convolution Kernels

In this section, the number of convolution kernels is changed to analyze the influence on the prediction performance. In the design of CNN, the numbers of two convolution layers are set to be the same in analyzing the influence of the number of convolution kernels. Table 6 shows the prediction results of 10-fold cross validation on the training set when *N*_*c*1_=*N*_*c*2_=4,8,16,32.

From Table 7, with the increase in number of kernels, the values of Sw and MCC show downward trend, and *N*_*c*1_=*N*_*c*2_=4 gets better prediction performance. Thus, the number of convolution kernel in conv1 is fixed on 4.

Then, we only change the number of convolution kernel in conv2.  Table 8 shows the prediction results when *N*_*c*2_=4,8,16,32. From Table 8, it obtains better Sw and MCC when *N*_*c*2_=4. Therefore, the parameters of conv1 and conv2 are set to 2 × 2 × 1 × 4 and 2 × 2 × 4 × 4, respectively.

### 3.6. Comparison with Other Methods

Our method is compared with other two state of the art methods IsUnstruct and ESpritz in this section.  Table 9 shows the prediction performance of three methods based on the test set. The prediction results of IsUnstruct and ESpritz are obtained by their respective network predictors. As shown in Table 9, our method gets the best Spec and similar Sens as ESpritz and thus obtains higher Sw and MCC.

## 4. Conclusions

In this paper, we propose a method to predict IDPs based on CNN and feature selection. Sequence properties and evolutionary properties are used to describe the differences between disordered residues and ordered residues. To highlight their specificity, sequence and evolutionary properties are preprocessed by 11 windows from length 7 to length 87, respectively. Then, the preprocessed features are combined into a feature matrix as the input of the prediction model. CNN can reflect the relationship between each feature and its neighboring features in the protein feature matrix and find out more information from different features and thus enrich the information proposed by protein sequences. Thus, we construct a CNN prediction model with two convolution layers and one fully connected layer, and each convolution layer is followed by a pooling layer. The parameters of each convolution kernel are set to 2 × 2 × 1 × 4 and 2 × 2 × 4 × 4, respectively. The simulation results show that the prediction performance of the proposed method gets better Sw and MCC than two competitive prediction methods IsUnstruct and ESpritz.

RETRACTED

## Figures and Tables

**Figure 1:** The structure of the CNN.

**Figure 2:** The prediction procedure of the proposed method.

**Figure 3:** The trend of each evaluation parameter with different number of windows.

**Table 1:** Datasets used in this paper.

Datasets	Disordered regions	Ordered regions	Disordered residues	Ordered residues
Training set	1,120	1,198	85,184	289,983
Test set	134	145	7,234	25,873
Total	1,254	1,343	92,418	315,856

**Table 2:** Prediction performance of different number of windows.

Step length	*N*_*win*_	Sens	Spec	Sw	MCC
1	25	0.8032	0.7594	0.5626	0.4852
2	13	0.7991	0.7676	0.5667	0.4909
3	9	0.8153	0.7676	0.5829	0.5038
4	7	0.8061	0.7787	0.5848	0.5089

**Table 3:** Prediction performance of different number of windows.

Window distance	*N*_*win*_	Sens	Spec	Sw	MCC
8	7	0.8061	0.7787	0.5848	0.5089
8	11	0.7833	0.8146	0.5979	0.5332
6	9	0.8153	0.7676	0.5829	0.5038
6	15	0.8914	0.7056	0.5970	0.5012

**Table 4:** Prediction performance of different convolutional layers.

Number of convolutional layers	The scale of convolutional parameter	Sens	Spec	Sw	MCC
2	3 × 3 × 1 × 8, 2 × 2 × 8 × 8	0.7833	0.8146	0.5979	0.5332
3	3 × 3 × 1 × 8, (2 × 2 × 8 × 8) × 2	0.7813	0.7961	0.5774	0.5092
4	3 × 3 × 1 × 8, (2 × 2 × 8 × 8) × 3	0.7654	0.7945	0.5599	0.4946
5	3 × 3 × 1 × 8, (2 × 2 × 8 × 8) × 4	0.7513	0.8028	0.5541	0.4932

**Table 5:** Prediction performance of different scales of convolution kernel in conv1.

The scale of conv1	Sens	Spec	Sw	MCC
2 × 2	0.7972	0.8090	0.6062	0.5373
3 × 3	0.7833	0.8146	0.5979	0.5332
4 × 4	0.7553	0.8414	0.5967	0.5457
5 × 5	0.7573	0.8377	0.5950	0.5423

**Table 6:** Prediction performance of different scales of convolution kernel in conv2.

The scale of conv2	Sens	Spec	Sw	MCC
2 × 2	0.7972	0.8090	0.6062	0.5373
3 × 3	0.7715	0.8291	0.6006	0.5422
4 × 4	0.7832	0.8047	0.5879	0.5210
5 × 5	0.8169	0.7734	0.5902	0.5114

**Table 7:** Prediction performance of different number of convolution kernel in conv1.

*N*_*c*1_, *N*_*c*2_	Sens	Spec	Sw	MCC
4	0.7960	0.8321	0.6281	0.5654
8	0.7972	0.8090	0.6062	0.5373
16	0.7442	0.8349	0.5791	0.5282
32	0.8226	0.7436	0.5660	0.4838

RETRACTED

**Table 8:** Prediction performance of different number of convolution kernel in conv1.

*N*_*c*1_, *N*_*c*2_	Sens	Spec	Sw	MCC
4	0.7960	0.8321	0.6281	0.5654
8	0.7972	0.8090	0.6062	0.5373
16	0.7442	0.8349	0.5791	0.5282
32	0.8226	0.7436	0.5660	0.4838

**Table 9:** Prediction performance of different number of convolution kernel in conv1.

Methods	Sens	Spec	Sw	MCC
Our method	0.7264	0.8301	0.5565	0.5060
IsUnstruct	0.7513	0.7855	0.5368	0.4711
ESpritz	0.7255	0.8135	0.5389	0.4840

## Data Availability

The datasets supporting the conclusions of this article are available on the DisProt database [24] (http://www.disprot.org/).

## Additional Points

In this paper, the authors add the technical details and experiments, improve the preprocessing process, retrain the prediction network, and improve the prediction performance.

## References

[1] Oldfield C. J., Uversky V. N., Kurgan L. (2019). Predicting functions of disordered proteins with MoRFpred. *Methods in Molecular Biology*.

[2] Peng Z., Xing Q, Kurgan L (2020). APOD: accurate sequence-based predictor of disordered flexible linkers. *Bioinformatics*.

[3] Hsu C. C., Buehler M. J., Tarakanova A. (2020). The order-disorder continuum: linking predictions of protein structure and disorder through molecular simulation. *Scientific Reports*.

[4] Van der Lee R., Buljan M., Lang B. (2014). Classification of intrinsically disordered regions and proteins. *Chemical Reviews*.

[5] Faustino A. F., Barbosa G. M., Silva M. (2019). Fast NMR method to probe solvent accessibility and disordered regions in proteins. *Scientific Reports*.

[6] Dunker A. K., Bondos S. E., Huang F., Oldfield C. J. (2015). Intrinsically disordered proteins and multicellular organisms. *Seminars in Cell & Developmental Biology*.

[7] Staneva I., Huang Y., Liu Z., Wallin S. (2012). Binding of two intrinsically disordered peptides to a multi-specific protein: a combined Monte Carlo and molecular dynamics study. *PLoS Computational Biology*.

[8] Midic U., Oldfield C. J., Dunker A. K., Obradovic Z., Uversky V. N. (2009). Protein disorder in the human diseasome: unfoldomics of human genetic diseases. *BMC Genomics*.

[9] Uversky V. N., Oldfield C. J., Dunker A. K. (2008). Intrinsically disordered proteins in human diseases: introducing the D2 concept. *Annual Review of Biophysics*.

[10] Oldfield C. J., Ulrich E. L., Cheng Y., Dunker A. K., Markley J. L. (2005). Addressing the intrinsic disorder bottleneck in structural proteomics. *Proteins: Structure, Function, and Bioinformatics*.

[11] Liu Y. (2017). A comprehensive review and comparison of existing computational methods for intrinsically disordered protein and region prediction. *Briefings in Bioinformatics*.

RETRACTED

[12] Prilusky J., Felder C. E., Zeev-Ben-Mordehai T. (2005). FoldIndex(C): a simple tool to predict whether a given protein sequence is intrinsically unfolded. *Bioinformatics*.

[13] Linding R. (2003). Globplot: exploring protein sequences for globularity and disorder. *Nucleic Acids Research*.

[14] Lobanov M. Y., Galzitskaya O. V. (2011). The Ising model for prediction of disordered residues from protein sequence alone. *Physical Biology*.

[15] Su C.-T., Chen C.-Y., Ou Y.-Y. (2006). Protein disorder prediction by condensed PSSM considering propensity for order or disorder. *BMC Bioinformatics*.

[16] Iqbal S., Hoque M. T. (2015). DisPredict: a predictor of disordered protein using optimized RBF kernel. *PLoS One*.

[17] Zhang T., Faraggi E., Xue B., Dunker A. K., Uversky V. N., Zhou Y. (2012). SPINE-D: accurate prediction of short and long disordered regions by a single neural-network based method. *Journal of Biomolecular Structure and Dynamics*.

[18] Walsh I., Martin A. J. M., Di Domenico T., Tosatto S. C. E. (2012). ESpritz: accurate and fast prediction of protein disorder. *Bioinformatics*.

[19] Liu Y. (2020). RFPR-IDP: reduce the false positive rates for intrinsically disordered protein and region prediction by incorporating both fully ordered proteins and disordered proteins. *Briefings in Bioinformatics*.

[20] Kozlowski L. P., Bujnicki J. M. (2014). MetaDisorder: a meta-server for the prediction of intrinsic disorder in proteins. *BMC Bioinformatics*.

[21] Fan X., Kurgan L. (2014). Accurate prediction of disorder in protein chains with a comprehensive and empirically designed consensus. *Journal of Biomolecular Structure and Dynamics*.

[22] Necci M., Piovesan D, Dosztányi Z, Tosatto S. C. E (2017). MobiDB-lite: fast and highly specific consensus prediction of intrinsic disorder in proteins. *Bioinformatics*.

[23] He H., Yang Y. Prediction of intrinsically disordered proteins with convolutional neural networks based on feature selection.

[24] Sickmeier M. (2007). DisProt: the database of disordered proteins. *Nucleic Acids Research*.

[25] He H., Zhao J. X. (2018). A low computational complexity scheme for the prediction of intrinsically disordered protein regions. *Mathematical Problems in Engineering*.

[26] Meiler J., Zeidler A., Schmschke F., Muller M. (2001). Generation and evaluation of dimension-reduced amino acid parameter representations by artificial neural networks. *Journal of Molecular Modeling*.

